# Machine Learning and Cloud-Based Knowledge Graphs to Recognize Suicidal Mental Tendencies

**DOI:** 10.1155/2022/3604113

**Published:** 2022-03-17

**Authors:** Vinit Kumar Gunjan, Y. Vijayalata, Susmitha Valli, Sumit Kumar, M. O. Mohamed, V. Saravanan

**Affiliations:** ^1^Department of Computer Science and Engineering, CMR Institute of Technology, Hyderabad, India; ^2^Department of CSE, GRIET, Telangana, India; ^3^Indian Institute of Management, Kozhikode, India; ^4^Mathematics Department, Zagazig University, Faculty of Science, Egypt; ^5^Department of Computer Science, College of Engineering and Technology, Dambi Dollo University, Dambi Dollo, Oromia Region, Ethiopia

## Abstract

To improve the quality of knowledge service selection in a cloud manufacturing environment, this paper proposes a cloud manufacturing knowledge service optimization decision method based on users' psychological behavior. Based on the characteristic analysis of cloud manufacturing knowledge service, establish the optimal evaluation index system of cloud manufacturing knowledge service, use the rough set theory to assign initial weights to each evaluation index, and adjust the initial weights according to the user's multiattribute preference to ensure that the consequences are allocated correctly. The system can help counselors acquire psychological knowledge in time and identify counselors with suicidal tendencies to prevent danger. This paper collected some psychological information data and built a knowledge graph by creating a dictionary and generating entities and relationships. The Han language processing word segmentation tool generates keywords, and CHI (Chi-square) feature selection is used to classify the problem. This feature selection is a statistical premise test that is acceptable when the chi-square test results are distributed with the null hypothesis. It includes the Pearson chi-square test and its variations. The Chi-square test has several benefits, including its distributed processing resilience, ease of computation, broad information gained from the test, usage in research when statistical assumptions are not satisfied, and adaptability in organizing information from multiple or many more group investigations. For improving question and answer efficiency, compared with other models, the BiLSTM (bidirectional long short-term memory) model is preferred to build suicidal tendencies. The Han language processing is a method that is used for word segmentation, and the advantage of this method is that it plays a key role in the word segmentation tool and generates keywords, and CHI (Chi-square) feature selection is used to classify the problem. Text classifier detects dangerous user utterances, question template matching, and answer generation by computing similarity scores. Finally, the system accuracy test is carried out, proving that the system can effectively answer the questions related to psychological counseling. The extensive experiments reveal that the method in this paper's accuracy rate, recall rate, and F1 value is much superior to other standard models in detecting psychological issues.

## 1. Introduction

Cloud manufacturing (CMfg) is a new service-oriented and knowledge-based networked and agile manufacturing model [1] that integrates advanced technologies, such as existing information technology, cloud computing [2], and the Internet of Things [3]. It centrally stores the optimized and integrated manufacturing resources in the cloud pool of the manufacturing system and provides users with various high-quality and fast manufacturing services on demand through the network. As a result, cloud manufacturing knowledge is a dynamic resource that is infiltrating all cloud manufacturing service life cycles [4]. At the same time, cloud manufacturing knowledge service (CMKS) is a knowledge transfer and sharing service that can effectively support cloud manufacturing. As a result, all manufacturing activities in the manufacturing environment are carried out efficiently, stably, and accurately.

The addition of knowledge services significantly improves cloud manufacturing systems' operational efficiency and problem-solving capabilities [5]. The organic combination of CMfg and knowledge services promotes the extension of “manufacturing as a service” to “knowledge as a service,” enabling enterprises to quickly obtain the required manufacturing knowledge and services with the support of the cloud platform, effectively solving the problems in the production and operation process of enterprises. Technical bottleneck problem improves its comprehensive competitiveness. It is a statistical premise test that is acceptable when the chi-square test results are distributed with the null hypothesis. It includes the Pearson chi-square test and its variations. The Chi-square test has several benefits, including its distributed processing resilience, ease of computation, broad information gained from the test, usage in research when statistical assumptions are not satisfied, and adaptability in organizing information from multiple or much more group investigations At present, scholars at home and abroad have explored the relevant theories and technologies of knowledge services in the cloud manufacturing environment. For example, author [6] proposed a personalized knowledge service technology based on user perception of the cloud manufacturing environment. The platform user task requirements and information actively push knowledge resources related to user manufacturing tasks. To a certain extent, it has promoted the evolution of cloud service platforms from “useable” to “easy to use.” Author [4] proposed a cloud manufacturing knowledge service method based on uncertain rule reasoning, which realizes the knowledge service from quantitative to qualitative and then from quantitative to qualitative. The conversion to quantitative provides a new idea for the accurate distribution of cloud manufacturing knowledge services. Reference [7] builds a knowledge service realization model for the machining process of blade parts in complex curved parts in a cloud manufacturing environment, which shortens the time to a certain extent. In this research, we have inferred that LSTM-based models are quite higher than ML algorithms because the LSTM framework for organizations was used to improve the knowledge graph, and a heuristics candidate answer ordering approach was employed to verify the system's performance.

The generation time of the tool path in the processing of blade parts is improved, and the processing efficiency and quality of the blade are improved. The literature [8] proposes an optimization method for matching the knowledge service demander and the provider and uses a fuzzy axiomatic design. The theoretical measurement of matching satisfaction provides a specific theoretical basis for matching the supply and demand of knowledge services. To realize the acquisition, storage, and sharing of different types of knowledge, literature [9] designs a cloud computing industry alliance based on the behavioral characteristics of knowledge interaction. To a certain extent, the knowledge resource sharing efficiency of the cloud computing industry alliance and the level of knowledge service have been improved. In this research, we have used the graph knowledge method. The limitation of this method is as follows: its evaluation measures concerning the model fit or factor levels cannot be done using graphic approaches since they do not provide certainty ranges for the variables (levels supplied by a correlation tool for all of this type of data are wrong). The above research has promoted the development of CMKS to a certain extent. The correctness and trustworthiness of the knowledge service offered cannot be ensured, resulting in low knowledge service performance. To that purpose, this study uses the user's mental behavioral traits as a judgment element, combining the benefits of the rough set theory in dealing with ambiguity and uncertainty. The CMKS is a knowledge-sharing and sharing service that can help cloud manufacturers succeed. As a consequence, all manufacturing operations in the manufacturing environment run smoothly, consistently, and precisely. Still, the research on the optimal decision-making method of knowledge service is relatively lacking. The accuracy and credibility of the provided knowledge service cannot be guaranteed, resulting in the low efficiency of knowledge service. To this end, this paper takes the user's psychological behavior characteristics as a decision-making factor and combines the advantages of the rough set theory in dealing with uncertainty and ambiguity. The optimal selection of services provides a reference idea and method.

## 2. Characteristics Analysis of Cloud Manufacturing Knowledge Service

CMKS is a kind of service guided by users' knowledge needs on the cloud manufacturing service platform, aiming at knowledge innovation, solving the manufacturing problems faced by users, and proactively providing users with personalized and specialized knowledge resources [10, 11]. The cloud manufacturing knowledge service (CMKS) is an information-sharing and sharing service that can help cloud manufacturers succeed. As a consequence, all manufacturing processes in the manufacturing environment run smoothly, consistently, and precisely. The integration of knowledge services enhances the operating effectiveness and problem-solving capacities of cloud manufacturing systems dramatically.

Compared with other services, knowledge services in the cloud manufacturing environment have the following salient features:

- Knowledge transformation is complex: there are many types of knowledge resources in the cloud manufacturing environment, including explicit knowledge, such as standards, patents, and documents, and tacit knowledge, such as experience and capabilities. Most of these highly personalized and challenging to standardize implicit knowledge resources come from different enterprises. Because of the inconsistency of knowledge resource management and processing methods, other users can benefit from the same knowledge resources. Therefore, converting cloud manufacturing knowledge service resources into their proper value is more challenging.
- Dynamic changes in value: in the cloud manufacturing environment, the value of complex manufacturing resources will decrease with aging and wear and tear, while the value of knowledge resources changes in different directions. For example, with the growth of age and the continuous accumulation of knowledge, the value of employee experience will become higher and higher. With the advancement of technology and users' higher requirements for product quality, the value of a specific method or patent will become higher. Cloud platforms need to monitor these knowledge resources and continuously update their value status to provide appropriate services to users at the right time.
- Highly integrated and shared: as an intellectual resource on the cloud manufacturing service platform, knowledge can provide oral, written, electronic, and other means and is minimally affected by geographical location. Therefore, compared with the complex manufacturing resources on the cloud manufacturing platform, the integration and sharing of resources are better.
- Heterogeneity and isomerism coexist: Because of the differences in thinking habits and problem-solving methods, the manifestations of knowledge condensed by people are also complex and diverse. The utility of the same type of knowledge services is also different. Therefore, knowledge services in the cloud manufacturing environment are heterogeneous.

## 3. Mental Illness

The pace of life in the current society is getting faster and faster, and people are facing more pressure from work and study, which makes them susceptible to mental illness. The new corona epidemic has brought psychological stress, panic, and anxiety to people and increased mental illnesses' prevalence. Mental diseases have become a significant global public health problem [12]. Mental illness requires timely treatment. Otherwise, the long-term accumulation of negative emotions it brings will cause incalculable consequences [13]. For example, Cui Yongyuan, the famous host of CCTV, suffered from depression because of his work troubles, and suicides of college and middle school students are also familiar [14].

On the one hand, this phenomenon is because of people's lack of basic knowledge of mental illness, lack of a clear understanding of the dangers of mental illness, and lack of advanced means to popularize the understanding of the mental illness. However, on the other hand, psychological counselors are in short supply, and counselors cannot get timely and effective help [15], lacking a scientific theoretical system to solve psychological problems intelligently. Therefore, an intelligent platform is needed to store the relevant psychological counseling knowledge. Then, when the user needs to obtain psychological understanding, the platforms can quickly get feedback from the immense ability to help and guide the mentally ill patients in time. The knowledge graph is a better method for intelligently storing information at present. This method was proposed by Google in 2012 and was quickly used for intelligent semantic search [16]. At present, artificial intelligence technology is gradually becoming mature and has penetrated all aspects of society, especially the development of natural language processing technology. The knowledge graph has more application prospects. The influence of social media on mental health is that it may have an effect on psychological health and behavioral activities that might have potential medical care concerns, and social networking holds an ever expanding route for both our everyday lives and globally. As a result, there is a pressing need to develop a better understanding of the long-term effects of social media on people's health. As an essential application direction of the knowledge graph, the question answering system based on knowledge graph can quickly find the correct answer from the knowledge graph through the input natural language question and present it to the user in the form of natural language, and this question answering system is efficient in response and feedback. To solve the above problems, this study, firstly, constructs a knowledge map of psychological counseling, promotes the knowledge of the mental illness, and provides quick psychological counseling services by establishing an immediate semantic psychological question answering system. The system uses the BiLSTM algorithm to detect suicidal tendencies, identify people who commit suicide, self-mutilation, and harm others in time, help users identify diseases, and help consultants understand relevant knowledge through knowledge quizzes. The BiLSTM method is used to predict the next piece of information based on the previous piece of information, making it ideal for having dealt with contextually related text data like sentences. As there might be delays of undetermined time across critical occurrences in a time series, LSTM methods are well-suited to categorizing, processing, and generating forecasts time series analysis. This research allows counselors to relieve their troubles, make up for the shortage of psychological counseling resources, and improve the work efficiency of psychological counseling.

## 4. Related Work

Knowledge graphs can be divided into general knowledge graphs and domain knowledge graphs. Typically available knowledge graph representatives include Freebase [8], DBpedia, Yago, Baidu, Google, etc., and they are mainly based on triple fact-based knowledge and have a certain tolerance for the quality of knowledge extraction. Typical domain knowledge graphs include e-commerce, finance, medical care, etc. In the field of e-commerce, take Alibaba as an example. Its knowledge graph has reached tens of billions, widely supporting commodity search, commodity shopping guides, intelligent question and answer, etc. Knowledge graphs allow investors and financiers to understand investment behaviors more quickly and grasp market conditions in the financial field. Aiming at the lack of financial charts, the author constructed a small financial knowledge graph using the crawled structured data, such as financial stocks and corporate information. At present, knowledge graphs are used primarily for clinical treatment decision support, medical intelligent semantic search, and medical question-answering systems in medicine. Clinical treatment decision support is to automatically generate a treatment plan for each patient according to the patient's situation, combine it with extensive data analysis in the medical field, and provide it to doctors for reference. Medical intelligent semantic search is to combine related entities from the medical knowledge graph. It can be used to query information such as the relationships and attributes to optimize the search results of medical information. Medical question and answer is another form of medical information retrieval. Its returned answers are in the form of natural language.

In terms of question answering system based on the knowledge graph, Tan Gang et al. used the LSTM model for entities/assertions to enhance the knowledge graph, used a heuristic candidate answer ranking method, and finally verified that the system has good performance through experiments. The author proposed a multi-round question answering system based on the knowledge graph of road regulations, which can better identify user intentions; the author with knowledge graph as database support, designed a question-and-answer system, which is based on the e-commerce field and realizes functions, such as question answering and reasoning. The authors are the parts of preprocessing, question classification, question template matching, and answer generation in a question answering system are implemented. The question answering procedures established above have been well-implemented in their respective fields, and the characteristics of the domain are integrated into the question answering system process. However, no scholars have studied question-answering systems in psychological counseling, and few texts have been classified as applied to question answering systems.

## 5. Question Answering System Framework

Compared with traditional search engines, the question answering system is more targeted, accurate, and more accessible for users to accept. The knowledge graph of psychological counseling realizes the association and integration of various kinds of knowledge in psychological counseling. It expresses understanding semantically in a professional and structured way, which can conveniently manage and query knowledge. The BiLSTM technique is used to predict suicidal inclinations, identify persons who commit suicide, self-mutilation, or damage others in a timely manner, assist users in identifying illnesses, and assist consultants in understanding necessary knowledge via knowledge assessments. The question-and-answer system constructed in this paper is biased toward acquiring professional knowledge of psychological counseling to help people with psychological problems find the correct answer and incorporate suicidal tendency detection to identify dangerous speeches promptly. The framework of the psychological counseling question answering system based on knowledge graph mainly includes four parts: data acquisition, graph construction, problem understanding, and user interface (Figure 1).

The data acquisition module of this system obtains relevant data of web pages through crawler technology. It combines the open data of Chat opera, organizes it into structured data through data processing, and uses Neo4j's python to drive py2neo to construct a knowledge graph. The question-understanding module uses the HanLP tool for word segmentation, part-of-speech tagging, etc. It then uses the CHI feature selection, uses the established BiLSTM model classifier to classify the question and judge whether it has suicidal tendencies, and finally uses the BERT (bidirectional encoder representation from transformers) model to convert queries into queries word vectors for semantic similarity calculation to match question templates and generate answers. The user interface module is the user's question input, and the system answers feedback and involves the mutual conversion of speech and text.

## 6. Question Answering System Implementation

### 6.1. Data Acquisition

The data sources for constructing knowledge graphs and classifying texts are web text data and Chat opera datasets, containing questions and label information. Web text data uses web crawler technology to crawl questions about suicide, self-injury, and injury tendencies and structured data about mental illnesses from Weibo Shudong, Baidu Know, 525 Psychology, Yixin, and Simple Psychology. Chat opera cooperated with some professionals to complete a corpus, which is the first open knowledge question-and-answer corpus in the field of psychological counseling, including 20,000 pieces of psychological counseling data. The dataset includes the annotation information of suicidal tendency, and the annotation information and question information are extracted from this dataset. Question information consists of three columns, cat-id, cat, and question, category (Table 1).

### 6.2. Knowledge Graph Construction

The knowledge graph is used as the database support of the question answering system. Hence, it is necessary to build the knowledge graph first. The primary purpose of constructing a knowledge map of psychological counseling, referring to the psychological counseling ontology database created by author [16] and consulting relevant scholars, is to analyze and summarize the psychological counseling process and the psychological knowledge involved. The psychological counseling information is divided into six categories: patients, symptoms, diagnostic criteria, causes of disease, diagnostic results, and treatment methods. Among them, disease causes are divided into biological causes, psychological causes, social causes, and defense mechanisms. There is a causal relationship between the cause of the disease and the diagnosis result. The diagnosis result is divided into the severity of the disease and the name of the mental illness. Diagnosis results and treatment methods are decisive, and treatment methods are divided into psychological treatment, drug treatment, and food treatment. The treatment method has an executive relationship with the patient. The patient needs to adopt the treatment method. The patient mainly includes the patient's identity information, such as age, height, occupation, gender, etc., and the patient's past medical history, which will affect the treatment of the consultant. There is a relationship between patients and symptoms, and symptoms mainly include severity and symptoms. Symptoms and diagnostic criteria are subordinate, and the diagnostic criteria include disease course criteria, severity criteria, and exclusion criteria. It shows that these elements involve various aspects of mental illness, and a question and answer usually involves parts of multiple aspects of mental illness. There are often causal relationships and dependencies between these elements. The protégé tool is used to build an entity-relationship diagram in the field of psychological counseling (Figure 2).

### 6.3. Instance Layer Construction

The crawled data is organized into structured data and is divided into 12 fields, which correspond to the entity-relationship of psychological counseling designed above, and they are divided into diseases and disease-related entities and attributes. The entities are diseases, aliases, symptoms, complications, drugs, and foods, and the details are susceptible populations, examination methods, treatment methods, cure periods, costs, and causes of disease.

The instance layer construction is divided into entity extraction, relation extraction, attribute extraction, triple construction, and knowledge storage. Here, the python-driven py2neo tool of the Neo4j tool is used to create the knowledge graph. Entity extraction is to extract entities according to the concept of the schema layer and save the entity field information in the structured data after sorting into a dictionary. Relation extraction finds the relationship between entities and saves the relationship between diseases and other entities and attributes as a dictionary. Attribute extraction is to extract the attribute information of some entities, i.e., to save the attribute field information in the sorted, structured data into a dictionary. The construction of triples is to organize the data into the form of (entity, relationship, entity), create nodes without attribute fields and disease nodes with attributes, and then use disease nodes as start-nodes and attribute nodes as end-nodes, with query = “match(p:%s), (q:%s), where p.name = “%s” and q.name = “%s” create(p)-[rel:%s{name: “%s”}]->(q)” % (start_node, end_node, p, q, rel_type, rel_name) command, and create a triple by creating a node relationship edge through the previously established relationship dictionary. Knowledge storage uses the platform to store the constructed knowledge graph. Here, the Neo4j platform stores the constructed small knowledge graph of psychological counseling Figure 3.

### 6.4. Word Segmentation Processing

Firstly, several mainstream word segmentation tools, such as Jieba, HanLP, and Chinese Academy of Sciences word segmentation NLPIR, are tested. The question-and-answer sentences of the psychological counseling QA corpus are selected as the data source. Before the test, psychology professionals were required to choose 100 data records and manually annotate them to achieve word segmentation and part-of-speech tagging as the actual value of the experiment. During the test, the 100 data records were processed with three-word segmentation tools, respectively, and the processing results were compared with the annotation results of professionals. The three-word segmentation tools obtained evaluation indicators, such as the accuracy rate, recall rate, F1 value, and word segmentation time (Table 2). Through the evaluation of the three-word segmentation tools, it can be concluded that NLPIR has the fastest word segmentation efficiency, however, HanLP has the highest accuracy. Combined with the evaluation results and psychological counseling needs, this study selected the HanLP tool for text segmentation. It imported the dictionary of disease information constructed above into HanLP's custom dictionary to make word segmentation more accurate.

### 6.5. Question Category

This paper combines the obtained psychological counseling question-and-answer data and consults professional psychological counselors to divide the frequently asked questions into five categories: disease identification, factual questions, method questions, list questions, and other questions. Disease identification questions mainly answer “what disease,” real questions mainly answer “what,” method questions mainly answer “how to do,” list questions mainly answer “what are,” and suicidal tendency questions are input by the user.

Since the principle of question classification is the same as that of suicidal tendency detection, the detailed process of suicidal tendency text classification is an example to illustrate. This article divides suicidal tendencies into four categories: suicidal tendencies, self-harm tendencies, harming others, and standard classes. Firstly, select 1500, 1200, 1000, and 9000 items from each dataset type as training data and then select another 150, 120, 100, and 900 items as test data. Then, using the HanLP word segmentation tool combined with stop words to perform word segmentation and afterword segmentation, the characteristic terms of suicidal tendency, self-harm tendency, injury tendency, and normal tendency were obtained, and the word cloud map of each category was drawn.

(1) $$\begin{array}{c} \text{chi}=\frac{n{\left(ad-bc\right)}^{2}}{\left(a+c\right)\left(b+d\right)\left(a+b\right)\left(c+d\right)}. \end{array}$$

Equation (1) is used to calculate the CHI value of all words after HanLP segmentation, which is used as the basis for feature selection of problem classification and suicidal tendency classification.

In the formula, *N* is the total number of labelled questions, *A* is the total number of documents used to record the word *t* in a specific category, *B* represents the documents that do not belong to a particular category but also contain the word *t*, and *C* represents a category that does not have the word *t*. In *t* documents, *D* represents documents that do not belong to a specific category and do not contain *t*. The CHI value denotes the degree of distinction between the two categories. The larger the CHI value, the more the word can represent a specific category.

Sort all the words according to the CHI value from large to small. Then, by selecting the 150 words with the most oversized CHI in each category, the selected 1000-dimensional feature list is obtained, and the feature vector weight of each question sentence is calculated, i.e., the word is in the question. If it appears in the sentence, it is assigned a value of 1. Otherwise, it is 0, and the final output is a feature vector that the classifier can recognize.

### 6.6. Problem Classification Model Selection

In text classification, five models of Naive Bayes, decision tree, SVM, XGBoost, and BiLSTM were used. Each model's training effects were compared, and the classification model with the best result was selected for the system. When testing each model, the precision rate, recall rate, and F1 value of each type of question will be obtained first, and then the precision rate, recall rate, and F1 value of all kinds of questions will be averaged. In the information extraction system, the BiLSTM model is tuned for suicidal propensity identification. The BiLSTM method is used to diagnose suicidal inclinations, identify those who commit suicide, self-mutilation, or damage others in a timely manner, assist users in identifying illnesses, and assist consultants in comprehending necessary facts through knowledge quizzes. Counselors can use this study to ease their stress, compensate for a lack of psychological treatment resources, and improve the efficiency of their job. In the information extraction system, the BiLSTM model is tuned for suicidal propensity identification. These values represent different models—the classification accuracy of (Table 3). From the test results in Table 3, it can be seen that the BiLSTM model is more accurate in the classification effect.

The BiLSTM model can predict the subsequent information using the previous information, which is suitable for dealing with contextually related text data, such as sentences. Taking the classification process of the BiLSTM model for suicidal tendency problems as an example, the HanLP word segmentation tool is selected for word segmentation, and the loss function and accuracy function image are obtained after the classification is completed (Figures 2–4).

In Figures 5–7, the train represents the training set. The test means the test set. The horizontal axis of the function is the number of training iterations, and the vertical axis represents the loss value and the accuracy value, respectively. When the number of iterations becomes more extensive, the loss rate gradually decreases and starts to level off when the number of iterations is 14. The training set tends to be between 0.1 and 0.2, and the test set tends to be between 0.2 and 0.3. The accuracy gradually increases and starts to level off when the number of iterations is 14. The training set tends to be 0.975, and the test set tends to be between 0.925 and 0.950.

By testing the precision rate, recall rate, and F1 value of each type of question to evaluate the model (Table 4), it can be concluded that the BiLSTM model has a better classification effect than the previous four models.

Comparing the questions answered correctly by the system with the questions answered incorrectly by the system, it can be seen that most of the questions answered correctly have similar characteristics to the question template, and some questions have the same entity and semantics as the question template. However, the expression methods are different, proving that the question answering system has a high semantic understanding ability. For questions that are not answered correctly, it has two characteristics: the system can recognize the entities in these questions but cannot recognize the semantic information that does not appear in the template, such as “What is the general age of onset of bipolar disorder?,” “Can bipolar disorder be cured?,” etc. Another feature is that the entity attribute information involved is not comprehensive enough, for example, what side effects of drugs exist and other attribute information should be added to the knowledge graph.

## 7. Conclusion

Today's society is facing the problem of knowledge explosion, especially the intermixing of knowledge in various fields, which affects people's acquisition and understanding of knowledge. This study is geared on gaining the professional understanding of psychological counseling to assist people with psychological issues in determining the proper answer, as well as including suicidal inclination detection to quickly identify risky remarks. The advantage of this research is that this study uses the user's psychological behavior traits as a decision-making element, combining the benefits of rough set theory in responding with uncertainty. A comparable notion and approach are provided by the best service choice. The vertical domain knowledge graph stores professional knowledge in a particular area, which significantly facilitates users to understand the knowledge in this field and use this knowledge to reduce losses or create a more excellent value. The psychological counseling knowledge graph and question answering system constructed in this paper has the following characteristics: (1) It provides a platform to store the knowledge of mental illness, which is more semantic than traditional databases. (2) The built question answering system realizes a complete set of word segmentation, question classification, question template matching, and answer generation, which can help users' judgmental illnesses and help users query relevant knowledge about mental illnesses research significance and value. (3) The BiLSTM model is optimized for suicidal tendency detection in the question answering system. The experimental results show that the accuracy rate, recall rate, and F1 value of the model in this paper are significantly better than other traditional models in the detection of suicidal tendency.

## Figures and Tables

**Figure 1:** The representative framework for psychological question answering system.

**Figure 2:** represents the accuracy of tendency classification model.

**Figure 3:** The F1-Score of tendency classification model.

**Figure 4:** Representation of the precision of the tendency classification model.

**Figure 5:** The accuracy of suicidal tendency classification by BiLSTM model.

**Figure 6:** The F1-Score of suicidal tendency classification by BiLSTM model.

**Figure 7:** Representation of the F1-Score of suicidal tendency classification by BiLSTM model.

**Table 1:** Examples of marked suicidal tendencies and normal questions.

Cat-id	Cat	Question
1	Tendency to self-harm	How to relieve the unreal feeling of depersonalization? In junior high school, my mood fluctuated a lot, and I cut myself with a knife because of some things and even suffered from severe depression
2	Normal	Ever since I reconciled with my boyfriend, he has always been hot and cold, and he does not want to admit that we are together. What does he mean?
3	Tendency to harm	Am I mentally ill? Ever since I was a child, I have had the idea of killing people and killing people around me.
0	Suicidal tendencies	I want to jump off a building, but I am afraid of heights

**Table 2:** Evaluation results of three-word segmentation tools.

Word segmentation tool	Accuracy	Recall	F1 value	Word segmentation time (s)
Jieba	0.90	0.89	0.89	12.480
HanLP	0.91	0.90	0.90	04.478
Academy of Sciences word segmentation NLPIR	0.81	0.75	0.78	30.0598

**Table 3:** Classification performance of model.

Model	Accuracy	F1-score	Precision
Naïve Bayes	79.65	80.56	69.56
Decision tree	74.52	81.26	65.25
SVM	75.62	76.85	70.62
XGBoost	80.54	82.54	72.56
BiLSTM	85.63	89.85	75.65

**Table 4:** Suicidal Tendency classification by BiLSTM Model.

Question	Accuracy	F1-score	Precision
Suicidal tendencies	81.26	79.56	75.62
Tendency to self-harm	82.62	80.54	85.61
Tendency to Hurt	85.68	84.56	90.25
Normal	95.62	97.56	98.56

## Data Availability

The data shall be made available on request.
